# Effects of *Artemisia annua* L. Essential Oil on Osteoclast Differentiation and Function Induced by RANKL

**DOI:** 10.1155/2022/1322957

**Published:** 2022-04-07

**Authors:** Wen Sun, Guangyue Yang, Fang Zhang, Chenguo Feng, Mingjie Liang, Pengfei Jia, Zhongliang Zhao, Hailing Guo, Yongfang Zhao

**Affiliations:** ^1^Shi's Center of Orthopedics and Traumatology, Shuguang Hospital Affiliated to Shanghai University of Traditional Chinese Medicine, Shanghai 201203, China; ^2^Institute of Traumatology and Orthopedics, Shanghai Academy of Traditional Chinese Medicine, Shanghai 201203, China; ^3^The Research Center of Chiral Drugs, Innovation Research Institute of Traditional Chinese Medicine, Shanghai University of Traditional Chinese Medicine, Shanghai 201203, China; ^4^Yuzhou Tianyuan Biotechnology Co., Ltd., Yuzhou 461000, China

## Abstract

**Objective:**

This study aimed to assess the main components of *Artemisia annua* L. essential oil (AEO) and determine their effect on the proliferation and differentiation of RAW264.7 cells induced by receptor activator for nuclear factor-ligand (RANKL) in vitro. Then, we tried to explain part of the function of its possible mechanisms.

**Materials and Methods:**

Essential oil was extracted from *Artemisia annua* L. Osteoclasts were induced *in vitro* by RANKL in mouse RAW264.7 cells. The experimental group was treated with different concentrations of AEO, while the control group was not treated with AEO. CCK8 was used to detect osteoclast proliferation. The osteoclasts were stained with TRAP. Western blot was used to detect protein in the MAPK pathway and the NF-*κ*B pathway after treatment with different concentrations of AEO. RT-PCR was used to determine the expression of osteoclast-related mRNA in cells.

**Results:**

The GC-MS analysis was used to obtain the main components of AEO, including camphor, borneol, camphor, borneol, terpinen-4-ol, p-cymene, eucalyptol, deoxyartemisinin, and artemisia ketone. The CCK8 results showed that the AEO volume ratio of 1 : 4000, 1 : 5000, and 1 : 6000 did not affect the proliferation of RAW264.7 cells. However, TRAP staining showed that AEO decreased osteoclast formation. Western blot results showed that the expression of protein TRAF6, p-p38, p-ERK, p-p65, and NFATc1 decreased in the MAPK pathway and the NF-*κ*B pathway affected by AEO. Furthermore, RT-PCR results showed that the expression of osteoclast resorption-related mRNAs (MMP-9, DC-STAMP, TRAP, and CTSK) and osteoclast differentiation-related mRNAs (OSCAR, NFATc1, c-Src, and c-Fos) also decreased in the experimental group.

**Conclusions:**

AEO inhibits osteoclast differentiation in vitro, probably by reducing TRAF6 activation, acting on the MAPK pathway and NF-*κ*B pathway, and inhibiting the expression of osteoclast-related genes.

## 1. Introduction

*Artemisia annua* L. belongs to the genus artemisia in Asteraceae and has a fragrance. The plant name has been checked on http://www.theplantlist.org mentioning the website's data. In the past, it was decocted with water to treat malaria, bone steaming hot flashes, summer heat, jaundice, etc. *Artemisia annua* L. contains monoterpenes (artemisia ketone, isoartemisia ketone, cineole, and camphor), sesquiterpenes (artemisinin, artemisinin A, artemisinin B, artemisinin C, and artemisia acid), and triterpenes (*β*-artemisinin acetate) [1]. Artemisinin is used as an anti-malarial drug for the clinical treatment of malaria. Artesunate may play a role in treating malaria, autoimmune diseases, cancer, diabetes, etc. [2]. Research on the effect of *Artemisia annua* L. on bone disease has gradually increased in recent years. Artesunate can reduce the level of inflammatory factors in the knee joint cavity [3], inhibit osteoclast secretion of axon guide factor netrin-1, and improve sensory nerve-mediated osteoarthritis pain [4]. It also inhibits the expression of vascular endothelial growth factors in fibroblast-like synovial cells of rheumatoid arthritis and has a therapeutic effect on synovitis [5]. An in vitro experiment showed that artemisinin and its derivatives could inhibit osteoclast differentiation [6].

Essential oil (EO) is a mixture of many chemical components in aromatic plants. EO is widely used as a perfume, food seasoning, and skincare product. It is also being developed in the pharmaceutical field since it has many pharmacological effects, such as antibacterial, anti-inflammatory, antioxidant, analgesia, and antitumor. For instance, EO has antibacterial activity against various Gram-positive and Gram-negative bacteria. Inhalation therapy with EO can treat sinusitis, acute and chronic bronchitis, and other diseases. Inhalation of EO can treat chronic illnesses that do not respond to conventional treatments, such as headaches, anxiety, depression, or epilepsy. Moreover, EO can improve the efficacy of various chemotherapeutic drugs, such as docetaxel. It can also enhance the immune system function of cancer patients [7].

*Artemisia annua* L. essential oil (AEO) combines aromatic volatile secondary metabolic molecules isolated from *Artemisia annua* L. by distillation. AEO has various effects, including antioxidation [8], antibacterial [9], anti-*α*-amylase, and anti-*α*-glucosidase [10]. Therefore, AEO can treat diseases caused by microbial drug-resistant infections, diabetes, and oxygen-free radicals. Monoterpenes are the most abundant compounds in essential oils. Paeoniflorin [11] found that monoterpenes suppress the proinflammatory cytokines in RAW 264.7 cells induced by lipopolysaccharide. Monoterpenes also suppress mitogen-activated protein kinase (MAPK) and nuclear factor-*κ*B (NF-*κ*B) signaling pathways. The MAPK and NF-*κ*B signaling pathways are essential in differentiating RAW264.7 into osteoclasts. Therefore, the active components of AEO can be further explored in different application fields. However, the AEO effect on osteoclast differentiation has not been elucidated.

The RAW264.7 cell line is mouse mononuclear macrophages and can be fused and differentiated into osteoclasts only via receptor activator for nuclear factor-*κ*B ligand (RANKL) [12, 13]. RANKL is a cytokine encoded by the tumor necrosis factor ligand family gene TNFSF11. It is an inducing factor for the differentiation and fusion of osteoclast precursors to form multinucleated osteoclasts [14]. It can bind to the receptor receptor activator for nuclear factor-*κ*B (RANK) on the surface of osteoclast progenitor cells and activate tumor necrosis factor-associated factor 6 (TRAF6) in the cells. TRAF6 activates some osteoclast-related pathways and cytokines [15] and can trigger the MAPK and NF-*κ*B pathways [16]. These pathways induce the expression and activation of nuclear factor of activated T-cell 1 (NFATc1), the main transcription factor of osteoclast differentiation [17, 18]. Transferring NFATc1 to the nucleus can promote the expression of genes related to osteoclast formation, thus enhancing osteoclast differentiation.

Herein, cellular and molecular biological methods were used to observe the effect of AEO on the proliferation and differentiation of RANKL-induced RAW264.7 cells. The possible mechanism of AEO inhibiting osteoclast differentiation by interfering with the RANKL signal pathway was also assessed. Therefore, this study may provide an experimental basis for preventing and treating metabolic osteopathy.

## 2. Materials and Methods

### 2.1. Reagents and Equipment

The following reagents and equipment were used: *Artemisia annua* L. essential oil (Yuzhou Tianyuan Biotechnology Co., Ltd., China), *n*-Alkenes (C8–C40) (AccuStandar, New Haven, USA), *n*-Hexane (Honeywell International Inc., Charlotte, USA), Anhydrous sodium sulfite (Shanghai Titan Scientific Co. Ltd., China), 5977B quadrupole mass spectrometer (Agilent Technologies, Santa Clara, USA), and fusion silica HP-5 MS capillary column (30 m × 0.25 mm × 0.25 *μ*m, Agilent Technologies).

The following were used: DMEM Culture medium (Sigma-Aldrich Cat: D6429), *α*-MEM Culture medium (Sigma-Aldrich Cat: M4655), RANKL (R & D Cat: CWA2519111), Fetal bovine serum (Gibco Cat: 10099141C), Penicillin Streptomycin (Gibco Cat: 15140122), CCK-8 (Biosharp Cat: BS350B), Trizol (Invitgen Cat: 15596018), Tartrate-resistant acid phosphatase Dyeing kit (Solarbio Cat: G1492), Prime Script RT Master Mix (Takara Ca: RR036A), TB Green Premix Ex Taq (TakaraCat: RR420A), RIPA (beyotime Cat: P0013B), Protease inhibitor (beyotime Cat: P1010), Phosphatase inhibitor (MedChemiExpress Cat: HY-K0021, HY-K0022, HY-K0023), BCA Protein Assay Kit (beyotime Cat: P0012), and Polyvinylidene Fluoride PVDF (beyotime Cat: FFP26).

The following were used: Carbon dioxide incubator (Heraeus), Enzyme-labeled instrument (BioTek synergy4), Microspectrophotometer (Thermo NanoDrop2000), PCR (Power Cycler), Real-time polymerase chain reaction system (Applied Biosystems), Optical microscope (Olympus IX71), and Western blot Gel analyzer (Bio-RAD).

### 2.2. Extraction of Essential Oil from *Artemisia annua L*

The leaves of *Artemisia annua* L. were collected, cleaned, and dried. Approximately 1 kg of the extract was extracted from dried leaves using petroleum ether (3 × 7 L). Organic extracts were combined, concentrated under reduced pressure, and then subjected to steam distillation at 100°C. Finally, the obtained mixture was separated using a separatory funnel, and the essential oil of the upper layer was collected (1∼2 mL).

### 2.3. Gas Chromatography-Mass Spectrometry (GC-MS) Analytical Conditions

The raw materials of essential oil from *Artemisia annua* L. were dried using anhydrous sodium sulfite before analysis. About 50 mg of dried oil was weighted and prepared in *n*-hexane at a 1 mg/mL concentration for sampling. The standard solution of *n*-alkenes was diluted in *n*-hexane to obtain a final testing concentration of 50 *μ*g/mL.

An Agilent 8860GC equipped with a 5977B quadrupole mass spectrometer was used for GC-MS analysis. A fused silica HP-5 MS capillary column was used to separate the components. Helium (purity >99.999%) was used as the carrier gas at a constant flow rate of 1.0 mL/min and a split ratio of 10 : 1. The oven temperature was as follows: an initial temperature of 50°C, ramped at 10°C/min to 120°C, at 1°C/min to 135°C, and then at 3°C/min to the final 240°C maintained for 8 min. The injection volume was 1 *μ*L. MS detection was conducted in the electron ionization (EI) mode (70 eV). The ion source, injector, and transfer line temperatures were 230°C, 250°C, and 250°C, respectively. MS analyzer was performed in the full scan mode (*m*/*z* 45–650), and the solvent delay time was set at 4 min. MassHunter GC-MS Data Acquisition (Version 10.0) and Qualitative Analysis (Version 10.0) were applied to control the equipment and acquire and treat raw data.

### 2.4. Cell Culture of Murine RAW264.7

RAW264.7 cells (Chinese Academy of Sciences TCM13) were cultured with DMEM complete culture medium containing 10% fetal bovine serum and 1% penicillin-streptomycin in CO2 incubator at 5% CO2, 37°C and saturated humidity.

RAW264.7 cells were inoculated in a culture plate with 5 × 10^3^ cells/cm^2^ when inducing osteoclast differentiation. After adhering to the plate, the cells were replaced by complete culture medium MEM and then induced with RANKL 50 ng/ml for five days. The culture medium was changed every two days.

### 2.5. Cell Counting Kit-8 (CCK-8) Proliferation Assay

RAW 264.7 cells were inoculated in a 96-well plate (2 × 10^3^ cells/well). After the cells were attached, different culture mediums were added to the experimental groups. The drug concentration (volume ratio 1 : 4000, 1 : 5000, 1 : 6000) with no statistical differences on cell survival rate was determined to assess the nontoxic effect of AEO on cells. The experimental group was treated with different concentrations of AEO and 50 ng/ml RANKL, while the control group was not treated with AEO. The CCK-8 staining solution (10 *μ*l) was added to each well at 0 h, 24 h, 48 h, 72 h, and 96 h after the intervention and then incubated for 2 h. The absorbance OD value of 450 nm was read using an enzyme labelling instrument, and cell activity was observed.

### 2.6. Tartrate-Resistant Acid Phosphatase (TRAP) Dyeing

Cells were inoculated in a 24-well plate (1 × 10^4^ cells / well) following the instructions of the TRAP staining kit and then treated. The experimental group was treated with 50 ng/ml RANKL and AEO (1 : 4000, 1 : 5000, 1 : 6000), while the control was not treated with AEO. Cells were stained after five days of intervention. The TRAP-positive cells with three or more nuclei in each well were counted.

### 2.7. Real-Time Quantitative Polymerase Chain Reaction (RT-PCR) Quantitative Analysis

RAW 264.7 cells were inoculated in a 6-well plate (5 × 10^4^ cells/well) and then treated. The experimental group was treated with 50 ng/ml RANKL and AEO (1 : 4000, 1 : 5000, 1 : 6000), while the control was not treated with AEO. AEO and RANKL were not added to the blank group. Total RNA was extracted using Trizol after 24 hours of cell culture. A spectrophotometer was used to quantify the mRNA, and 1 *μ*m RNA was reverse transcribed into cDNA via PCR. Forty cycles of two-step polymerase chain reaction amplification were performed on the Applied Biosystems real-time polymerase chain reaction system (95°C 5 s, 60°C 30 s) using the TB Green Premix Ex Taq kit. The primer sequence was as follows: GAPDHA-F: AGGTCGGTGTGAACGGATTTG, GAPDHA-R: GGGGTCGTTGATGGCAACA, MMP9-F: GACGACATAGACGGCATCC, MMP9-R: TGGTTCAGTTGTGGTGGTG, DC-STAMP-F: TCCTCCATGAACAAACAGTTCCAA, DC-STAMP-R: AGACGTGGTTTAGGAATGCAGCTC, TRAP-F: AAATCACTCTTCAAGACCAG, TRAP-R: TTATTGAACAGCAGTGACAG, CTSK-F: GGGAGAAAAACCTGAAGC, CTSK-R: ATTCTGGGGACTCAGAGC, c-Src-F: CCAGGCTGAGGAGTGGTACT, c-Src-R: CAGCTTGCGGATCTTGTAGT, OSCAR-F: CCTAGCCTCATACCCCCAG, OSCAR-R: CGTTGATCCCAGGAGTCACAA, NFATc1-F: GGAGAGTCCGAGAATCGAGAT, NFATc1-R: TTGCAGCTAGGAAGTACGTCT, c-Fos-F: GCGAGCAACTGAGAAGAC, c-Fos-R: TTGAAACCCGAGAACATC. The mRNA level of the target gene was normalized to the mRNA level of GAPDH.

The ΔCt (Ct target gene-Ct GAPDH) and −ΔΔCt (ΔCt mean −ΔCt) were calculated, and 2^−ΔΔCt^ was used to express the analyzed genes.

### 2.8. Western Blot Analysis

RAW 264.7 cells were inoculated in a 6-well plate (5 × 10^4^ cells/well) and then treated. The experimental group was treated with 50 ng/ml RANKL and AEO (1 : 4000, 1 : 5000, 1 : 6000), while the control was not treated with AEO. Similarly, AEO and RANKL were not added to the blank group. Cells were collected using RIPA lysate containing 1% protease and 5% phosphatase inhibitors and then centrifuged at 4°C, 12000*g* for 20 min. Proteins (20 ug) were separated on 10% SDS-polyacrylamide gel by electrophoresis. The separated proteins were then imprinted on the PVDF membrane, blocked with 5% skim milk for 1 h, and then incubated with the appropriate dilution of the first antibody at 4°C overnight. The membrane was washed with TBST buffer containing 0.05% tween-20 and then incubated with HRP labelled secondary antibodies for 1 h. The membrane was washed using TBST, and the target protein band was obtained via a gel analyzer. The grey level of the band was analyzed using Image J, and the relative protein expression was calculated via the normalization of the actin protein. The following primary antibodies were used: Anti-rabbit *β*-actin (1 : 1000, Cell Signaling Technology Cat : 3700), anti-rabbit p-p38 (1 : 1000, Cell Signaling Technology Cat : 4511), anti-rabbit p-ERK (1 : 1500, Cell Signaling Technology Cat : 4370), anti-rabbit TRAF6 (1 : 1000, Abcam Cat : ab33915), anti-mouse PCNA (1 : 1000, Abcam Cat : ab29), anti-rabbit NFATc1 (1 : 1500, Biomake Cat : A5784), and anti-rabbit I*κ*B-*α* (1 : 1500, Biomake Cat : A5599). HRP-labelled goat anti-rabbit (1 : 10000, Proteintech Cat : SA00001-1) and goat anti-mouse IgG (1 : 10000, Proteintech Cat : SA00001-1) were used as secondary antibodies.

### 2.9. Statistical Analysis

All data were expressed as mean ± standard deviation (SD). A single-factor analysis of variance (ANOVA) was used for multiple comparisons. *P* < 0.05 was considered the statistically significant level. The quantitative data of TRAP-positive cells represented six experiments in each group, while all the PCR and WB experiments data represented three groups. GraphPad Prism9 software (GraphPad Software Inc.) was used for all statistical mapping analyses.

## 3. Results

### 3.1. Qualitative Analysis of Essential Oil via GC-MS

NIST Mass Spectral Library search identified the components of AEO. Further identification was confirmed by comparing their retention indices with data from the literature. The typical total ion chromatography obtained from the GC-MS analysis is presented in Figure 1. Fifty-one volatile compounds were identified using the mass spectrum search and retention index, and the main volatile components were terpenoids, including camphor, borneol, eucalyptol, and piperitone. The name, retention time, CAS number, and the retention index (from experiments and literature) of each volatile compound identified from the AEO are shown in Table 1.

### 3.2. Effect of AEO on the Proliferation of RANKL-Induced RAW264.7 Cells

RAW264.7 cells were fused and differentiated into osteoclasts (Figure 2(a)) after induction with RANKL for five days. The expansion of RANKL-induced RAW264.7 cells accelerated and slowed after 72 h (Figure 2(b)). Cell survival rates in the experimental group were higher than 90% after 24 h, 48 h, 72 h, and 96 h of intervention. Furthermore, cell survival rates in the experimental and control groups were not statistically different (Figure 2(c)). Western blot did not show significant differences in PCNA (proliferating cell nuclear antigen) between the experimental and control groups (Figure 2(d)). Therefore, there was no inhibitory effect on cell proliferation at the concentration of 1 : 4000, 1 : 5000, and 1 : 6000.

### 3.3. AEO Inhibits Osteoclast Resorption-Related Protein Expression

TRAP staining showed that almost no osteoclasts were observed when the concentration was 1 : 4000 and 1 : 5000, while a few osteoclasts formed when the concentration was 1 : 6000 (Figures 3(a) and 3(b)).

RT-PCR showed that the osteoclast bone resorption-related protein matrix metalloproteinase-9 (MMP-9) mRNA expression more significantly decreased after the AEO intervention (1 : 4000, 1 : 5000 and 1 : 6000) than in the control group. The terms of the osteoclast bone resorption-related protein dendritic cell-specific transmembrane protein (DC-STAMP) mRNA, the osteoclast specific marker enzyme cathepsin K (CTSK), and TRAP [19] were lower in the experimental group than in the control group. However, the expression was not significantly different among the three experimental groups (Figure 3(c)). Therefore, these results show that AEO inhibits the number of osteoclasts in a dose-dependent manner. AEO also inhibits the expression of osteoclast-related specific mRNA.

### 3.4. AEO Inhibits the RANKL-Induced p-38/MAPK, ERK/MAPK, and NF-*κ*B Pathways in RAW264.7 Cells

Western blot showed that TRAF6 decreased significantly after AEO intervention at 1 : 4000 than in the control group, while it was not different between the 1 : 5000 and 1 : 6000 groups. TRAF6 was lower in the 1 : 4000 group than in the 1 : 5000 and 1 : 6000 groups (Figure 4(a)). The amount of NFATc1 was significantly decreased after AEO intervention at 1 : 4000, 1 : 5000, 1 : 6000 than in the control group. NFATc1 was lower in the 1 : 4000 group than in the 1 : 5000 and 1 : 6000 groups (Figure 4(b)). Phosphorylation of extracellular signal-regulated kinase (ERK) and p38 in the MAPK subfamily can promote osteoclast differentiation and prolong survival time [20]. The amount of p-p38 protein decreased significantly after AEO intervention at 1 : 4000 than in the control group. The amount of p-p38 significantly reduced in the 1 : 4000 group than in the 1 : 6000 group in a dose-dependent manner (Figure 4(c)). The amount of p-ERK significantly reduced in the 1 : 4000 group than in the control group, while it increased in the 1 : 6000 group. However, p-ERK was not different among the three experimental groups (Figure 4(d)).

Therefore, AEO has different effects at various concentrations on the content of TRAF6, p-p38, p-ERK, and NFATc1 proteins. Herein, AEO (1 : 4 000) was used to detect cell protein for 24 h, 48 h, 72 h, and 96 h. The results showed that the protein contents of TRAF6, p-p38, p-ERK, and NFATc1 were not significantly different in cells treated with AEO for 24 hours and in the control group. However, the protein of TRAF6, p-p38, p-ERK, and NFATc1 decreased at 48 h, 72 h, and 96 h (Figure 4(e)).

The activation of the NF-*κ*B pathway can produce NF-*κ*B/RelA [21], such as NF-*κ*B p65. The degradation of I*κ*B*α* (I-kappa-B kinase alpha) can transfer NF-*κ*B to the nucleus to promote the transcription of the target gene. The amount of I*κ*B*α* protein decreased significantly in the control group. However, I*κ*B*α* increased after AEO intervention than in the control group (Figure 5(a)). Compared to the control group, there was no significant increase of I*κ*B*α* in the experimental groups at 24 h, 48 h, 72 h, and 96 h (Figure 5(b)). The amount of p-p65 protein decreased significantly in the 1 : 4000 group compared to the control group. There is no significant difference of p-p65 in the 1 : 4000 group between the 1 : 5000 and 1 : 6000 group (Figure 5(c)). Similar results also found that the protein of p-p65 decreased at 48 h, 72 h, and 96 h after AEO intervention (Figure 5(d)).

The RT-PCR results showed that the mRNA levels of osteoclast differentiation-related protein NFATc1 were significantly downregulated in the experimental group than in the control group (Figure 6). The translocation of NFATc1 to the nucleus can promote the mRNAs expression of osteoclast formation-related genes, such as neuronal proto-oncogene tyrosine-protein kinase Src (c-Src), osteoclast-associated immunoglobulin-like receptor (OSCAR), and cellular oncogene Fos (c-Fos). In this article, the level of c-Src mRNA expression was lower in the 1 : 4000 group than in the 1 : 6000 group. The mRNA expression level of OSCAR was lower in the 1 : 4000 group than in the 1 : 5000 group. However, the mRNA levels of NFATc1 and c-Fos were not significantly different among the three experimental groups. Therefore, these results show that AEO inhibits osteoclast differentiation-related pathways and mRNA expression.

## 4. Discussion

Herein, AEO inhibited osteoclast formation. It also reduced the expression of osteoclast marker proteins by reducing the activation of TRAF6, inhibiting the p38/MAPK and ERK/MAPK pathways, and reducing NFATc1 synthesis (Figure 7). These results suggest that AEO inhibits osteoclast differentiation.

Osteoclasts decompose the collagen matrix during bone metabolism to form bone lacunas by secreting acid hydrolase [22]. In addition, osteoblasts form new bone to fill bone lacunae to maintain bone homeostasis. The imbalance of bone homeostasis may lead to metabolic bone diseases, such as osteoporosis [23] and periodontitis [24]. The function of osteoclasts is also closely related to the immune system. The number and activity of osteoclasts increase in inflammatory diseases, such as rheumatoid arthritis and Crohn's disease [25, 26]. Mature multinucleated osteoclasts are formed via proliferation, migration, cell adhesion, and fusion of progenitor cells [27]. Therefore, it is necessary to control the number and activity of osteoclasts to reduce bone loss and inhibit joint inflammatory diseases. Thus, negative regulation of osteoclast differentiation induced by RANKL can regulate bone metabolism and prevent or treat metabolic osteopathy.

GC-MS analysis showed that monoterpenes are the main substances in AEO, such as camphor, borneol, terpinen-4-ol, p-cymene, eucalyptol, deoxyartemisinin, and artemisia ketone. Sourav Das [9] also found camphor, terpinen-4-ol, and other active components in different formulations of AEO. Santomauro [28] and Zhigzhitzhapova [8] extracted camphor, *α*-pinene, and 1,8-cineole from AEO. The chemical composition of AEO extracted by Jaradat [10] is mainly borneol, bornyl acetate. The above findings are consistent with this analysis. Individual differences in the substances extracted from AEO may be due to the plants' geographical location, climate, and harvest time.

Camphor is the main component of many aromatic plant essential oils. It has anti-inflammatory and analgesic properties [29]. Dr. Duke's Phytochemical Databases and Ethnobotanical Databases (https://www.ars-grin.gov/duke/) show that *Artemisia annua* contains camphor (concentration in the leaves, 6460 ppm). Borneol and its derivatives have antibacterial, anti-inflammatory, antiviral, antiproliferation, and antiedema effects [30]. They can also relieve mild muscle and joint pain caused by arthritis or sprain [31]. Brand [32] showed that terpinen-4-ol could inhibit t inflammation via lipopolysaccharide-stimulated monocytes. Eucalyptol controls airway mucus hypersecretion and asthma by inhibiting anti-inflammatory cytokines [33]. Zhong [29] found that p-cymene can significantly inhibit the activation of EKR, p38, and c-Jun N-terminal kinases in RAW 264.7 cells by reducing proinflammatory cytokines. The AEO monoterpenes, such as p-cymene, can also minimize osteoclast differentiation.

We found that AEO inhibited the differentiation of RAW264.7 cells into osteoclasts induced by RANKL. As a shared signal sensor of TNF, Toll-like/IL-1, and the cellular inflammatory receptor family, TRAF6 is located upstream of the MAPK and NF-*κ*B pathway [34]. The MAPK and NF-*κ*B pathways play an essential role in osteoclast differentiation. MAPK pathway includes p38, JNK, and ERK pathways. Western blot images show that TRAF6 protein increased significantly after RANKL-induced RAW264.7 cells, and it increased with the induction time, consistent with other studies [35,36]. An *in vitro* experiment [6] showed that artemisinin and its derivatives could decrease the amount of TRAF6 protein and inhibit the activation of TRAF6 recruitment in RAW264.7 cells. In this paper, the amount of intracellular TRAF6 protein decreased after the AEO intervention.

Furthermore, the proteins p-p38 and p-ERK in the MAPK pathway increased significantly after RANKL induction and increased with induction time. A study has shown that Dihydroartemisinin in *Artemisia annua* L. inhibits RANKL-induced ERK phosphorylation of Pathways [37]. We also observed that p-p38 and p-ERK protein decreased after the AEO intervention. The AEO could inhibit the phosphorylation of p38 and ERK in a dose-dependent manner. The main transcription factor of osteoclast differentiation, NFATc1, began to accumulate and increase after 24 h–48 h after induction [38], similar to our western blot results. In western blot images, AEO can inhibit NFATc1 in a dose-dependent manner. The ability to inhibit NFATc1 is an integral part of the mechanism of AEO that inhibits osteoclast formation induced by RANKL. The NFAT signal is located downstream of the MAPK pathway and downstream of the NF-*κ*B pathway. AEO may be also achieved by suppressing the NF-*κ*B signal by suppression of NFATc1.

The RANKL-induced NF-*κ*B pathway is an important signal pathway activated during osteoclast formation. The interaction between RANK and RANKL results in proteasome degradation of I*κ*Ba, followed by the release of NF-*κ*B/RelA dimers, such as NF-*κ*B p65, which are then transported from the cytoplasm to the nucleus to initiate osteoclast-specific gene transcription [39–41]. In the previous studies, Artesunate and Dihydroartemisinin inhibited the activation of NF-*κ*B and osteoclast formation induced by RANKL by regulating the degradation of I*κ*B*α* protein and the expression of downstream genes in vitro [37, 42]. The effect of AEO on the NF-*κ*B pathway is yet to be reported. Results show that AEO inhibits the phosphorylation of NF-*κ*B p65 and the degradation of I*κ*B*α*, thus inhibiting the activation of NF-*κ*B induced by RANKL. AEO can also inhibit osteoclast differentiation by inhibiting the NF-*κ*B pathway.

AEO decreased the expression of osteoclast-related gene mRNA, including c-Fos, c-Src, and OSCAR, thus reducing osteoclast differentiation. The c-Fos is located downstream of MAPK and can form a close nuclear phosphoprotein with Jun/AP-1 transcription factors, essential for bone cell development and maintenance. Kinase c-Src can phosphorylate the tyrosine residues of c-Fos [43]. The OSCAR is an immunoglobulin-like receptor associated with osteoclast differentiation [44]. As a costimulatory signal needed for RANKL-mediated activation of NFATc1, OSCAR is the direct target of NFATc1 [40]. Therefore, the mRNA expression of c-Src, c-Fos, and OSCAR in cells can reflect the formation mechanism of osteoclasts.

AEO also decreased the expression of DC-STAMP, MMP-9, TRAP, and CTSK, thus decreasing the bone resorption function of osteoclasts. After RANKL stimulation, the DC-STAMP moves from the surface of osteoclast progenitor cells to the cytoplasm [45], which is one of the fusion mediators directly regulated by NFATc1 [36]. DC-STAMP is related to bone resorption and osteoclast fusion and participates in TRAP expression in osteoclast precursors [46, 47]. MMP-9 is associated with the migration of RAW264.7 cells [48]. The CTSK and TRAP are specific markers of osteoclasts [19]. Besides, the mRNA expression of CTSK, TRAP, MMP-9, and DC-STAMP genes can reflect the bone resorption function of osteoclasts.

Therefore, the differentiation of mouse osteoclasts is inhibited by AEO *in vitro*. Besides, this study can provide insights into preventing and treating metabolic bone diseases. However, the effect of AEO on osteoclast differentiation has not been tested *in vivo*. The specific mechanism of AEO deserves further exploration.

## 5. Conclusions

These results suggest that AEO can inhibit osteoclast formation and bone resorption by inhibiting RANKL-induced activation of the MAPK pathway and the NF-*κ*B pathway *in vitro*.

## Figures and Tables

**Figure 1:** GC-MS spectrum of artemisia essential oil. The compounds were identified using the NIST library and their corresponding mass spectrum fragmentation pattern.

**Figure 2:** Effect of AEO on the proliferation of RANKL-induced RAW264.7 cells. (a) RAW264.7 cells and RANKL-induced osteoclasts (200x). (b) RAW264.7 cell growth curve. (c) Effects of different concentrations of AEO on cell survival at 24 h, 48 h, 72 h, and 96 h. (d) The expression of PCNA protein in cells treated with AEO (^*∗*^*P* < 0.05 VS. control). Data represented three experiments in each group.

**Figure 3:** AEO inhibits osteoclast differentiation. (a) The number of osteoclasts at different concentrations of AEO. The quantitative data of TRAP-positive cells represented six experiments in each group. (b) TRAP staining showing multinucleated cells treated with different concentrations of AEO (200x). (c) The expression of osteoclast-associated mRNA (MMP-9, DCSTAMP, TRAP, CTSK) (^∧^*P* < 0.05 VS. blank; ^*∗*^*P* < 0.05 VS. control; ^#^*P* < 0.05 VS. 1 : 4000; ^+^*P* < 0.05 VS. 1 : 5000). Data represented three experiments in each group.

**Figure 4:** Mechanism of AEO inhibiting osteoclast differentiation. (a–d) The expression of Traf6, NFATc1, p-p38, and p-ERK after AEO intervention. (e) Expressions of Traf6, NFATc1, p-p38, and p-ERK after AEO intervention (1 : 4000) for 24 h, 48 h, 72 h and 96 h (^^^*P* < 0.05 VS. blank; ^*∗*^*P* < 0.05 VS. control; ^#^*P* < 0.05 VS. 1 : 4000; ^+^*P* < 0.05 VS. 1 : 5000). Data represented three experiments in each group.

**Figure 5:** The effect of AEO on I*κ*B*α*, p-p65 protein. (a) The expression of I*κ*B*α* after AEO intervention. (b) The expression of I*κ*B*α* protein after 24 h, 48 h, 72 h and 96 h of AEO intervention. (c) The expression of p65 and p-p65 after AEO intervention. (d) The expression of p65 and p-p65 protein after 24 h, 48 h, 72 h and 96 h of AEO intervention (^^^*P* < 0.05 VS. blank; ^*∗*^*P* < 0.05 VS. control). Data represented three experiments in each group.

**Figure 6:** AEO decreased the expression of mRNA (OSCAR, NFATc1, c-Src, c-FOS) associated with osteoclast differentiation (^^^*P* < 0.05 VS. blank; ^*∗*^*P* < 0.05 VS. control; ^#^*P* < 0.05 VS. 1 : 4000). Data represented three experiments in each group.

**Figure 7:** The mechanism diagram of AEO in vitro on osteoclast differentiation. AEO reduced TRAF6 activation and inhibited ERK and p38 phosphorylation. AEO also inhibits the phosphorylation of NF-*κ*B p65 and the degradation of I*κ*B*α*.

**Table 1:** Chemical composition of AEO.

Peak no.	Retention time (min)	Matched compound in the NIST database	CAS no.	Retention index (HP-5 MS)	
				RI_exp_	RI_lit_
1	6.861	Methyl hexanoate	106-70-7	922	924
2	7.377	Camphene	79-92-5	956	954
3	7.968	Trans-5-isopropenyl-2-methyl-2-vinyltetrahydrofuran	54750-70-8	995	994
4	8.509	P-cymene	99-87-6	1027	1025
5	8.662	Eucalyptol	470-82-6	1036	1035
6	9.069	Artemisia ketone	546-49-6	1059	1061
7	9.667	Dehydro-p-cymene	1195-32-0	1094	1095
8	10.990	Camphor	76-22-2	1152	1150
9	11.448	Borneol	507-70-0	1172	1172
10	11.703	Terpinen-4-ol	562-74-3	1183	1182
11	12.021	*α*-Terpineol	98-55-5	1197	1198
12	12.765	Cis-carveol	1197-06-4	1221	1221
13	13.980	Piperitone	89-81-6	1258	1257
14	14.585	Methyl 3-phenylpropionate	103-25-3	1276	1279
15	18.173	Cis-carvyl acetate	1205-42-1	1368	1365
16	18.917	Copaene	3856-25-5	1386	1379
17	19.643	Jasmone	488-10-8	1405	1403
18	20.412	Caryophyllene	87-44-5	1433	1432
19	24.859	*δ*-Cadinol	19435-97-3	1649	1646
20	29.873	Deoxyartemisinin	72826-63-2	2080	2058

## Data Availability

The data used to support the findings of this study are included within the article.

## Abbreviations

AEO: *Artemisia annua* L. essential oil
EO: Essential oil
RANK: Receptor activator for nuclear factor-*κ*B
RANKL: Receptor activator for nuclear factor-ligand
MAPK: Mitogen-activated protein kinase
p-ERK: Extracellular signal-regulated kinase
TRAF6: Tumor necrosis factor-associated factor 6
NFATc1: Nuclear factor of activated T-cell 1
GC-MS: Gas chromatography-mass spectrometry
CCK8: Cell counting kit-8
TRAP: Tartrate-resistant acid phosphatase
RT-PCR: Real-time quantitative polymerase chain reaction
PCNA: Proliferating cell nuclear antigen
MMP-9: Matrix metalloproteinase-9
DC-STAMP: Dendritic cell-specific transmembrane protein
CTSK: Cathepsin K
NF-*κ*B: Nuclear factor kappa B
I*κ*B*α*: I-kappa-B kinase alpha
OSCAR: Osteoclast-associated immunoglobulin-like receptor
c-Src: Neuronal proto-oncogene tyrosine-protein kinase src
c-Fos: Cellular oncogene Fos.
